The article "Static compression down-regulates N-cadherin expression and facilitates loss of cell phenotype of nucleus pulposus cells in a disc perfusion culture" was retracted in 2024. Reasons: duplicated images; compromised peer review; concerns about the authorship.

# Static compression down-regulates N-cadherin expression and facilitates loss of cell phenotype of nucleus pulposus cells in a disc perfusion culture

**DOI:** 10.1042/BSR20171551

**Published:** 2018-02-08

**Authors:** Haibo Zhou, Jianmin Shi, Chao Zhang, Pei Li

**Affiliations:** 1 Department of Orthopedic Surgery, The First Affiliated Hospital of Wenzhou Medical University, Wenzhou, Zhejiang 325000, China; 2 Department of Orthopedic Surgery, Liaocheng People’s Hospital and Liaocheng Clinical School of Taishan Medical University, Liaocheng, Shandong 252000, China; 3 Department of Orthopedic Surgery, No. 89 Hospital of PLA, Weifang, Shandong 261026, China

**Keywords:** compression, degeneration, nucleus pulposus, N-cadherin, organ culture

## Abstract

Mechanical compression often induces degenerative changes of disc nucleus pulposus (NP) tissue. It has been indicated that N-cadherin (N-CDH)-mediated signaling helps to preserve the NP cell phenotype. However, N-CDH expression and the resulting NP-specific phenotype alteration under the static compression and dynamic compression remain unclear. To study the effects of static compression and dynamic compression on N-CDH expression and NP-specific phenotype in an *in vitro* disc organ culture. Porcine discs were organ cultured in a self-developed mechanically active bioreactor for 7 days and subjected to static or dynamic compression (0.4 MPa for 2 h once per day). The noncompressed discs were used as controls. Compared with the dynamic compression, static compression significantly down-regulated the expression of N-CDH and NP-specific markers (laminin, brachyury, and keratin 19); decreased the Alcian Blue staining intensity, glycosaminoglycan and hydroxyproline contents; and declined the matrix macromolecule (aggrecan and collagen II) expression. Compared with the dynamic compression, static compression causes N-CDH down-regulation, loss of NP-specific phenotype, and the resulting decrease in NP matrix synthesis.

## Introduction

Intervertebral disc (IVD) degeneration (IDD) is a common cause of low back pain (LBP) [1]. As a debilitating condition, LBP leads to substantial socioeconomic loss and brings a heavy burden to the healthcare system [2]. Because the traditional treatments (i.e. conservative therapy or surgical therapy) mainly aim to symptom alleviation, several kinds of new strategies are being developed to biologically regenerate the degenerative disc tissues [3]. Nevertheless, it will take a long time to get exciting breakthroughs.

The IVD plays an important role in the biomechanics of the spine [4]. It participates in load bearing, absorption, and transmission between two adjacent vertebral bones [4]. During daily activities, the IVDs experience various and complex mechanical stimuli. Amongst these mechanical loads, the static compression or dynamic compression has been usually applied in the research field of disc degeneration [5–7]. Though a general consensus has been reached that the dynamic compression is more physiologically relevant than the static compression *in vivo* [7], and that the static compression often causes negative effects on healthy disc biology compared with the dynamic compression [6], the potential mechanisms need to be further studied.

The article "Static compression down-regulates N-cadherin expression and facilitates loss of cell phenotype of nucleus pulposus cells in a disc perfusion culture" was retracted in 2024. Reasons: duplicated images; compromised peer review; concerns about the authorship.

N-cadherin (N-CDH) is a calcium-dependent adhesion molecule [8,9]. Previously, several studies have showed that N-CDH is a cellular maker of healthy and normal disc nucleus pulposus (NP) cells [10,11]. Notably, N-CDH-mediated signaling is beneficial to maintain NP phenotype and the resulting NP matrix biosynthesis [12,13]. In light of the positive role of N-CDH in keeping normal NP cell phenotype and the relatively negative effects of static compression on NP matrix remodeling compared with the dynamic compression, we deduce that N-CDH-mediated signaling may be correlated with the static compression-induced unfavorable effects on disc NP biology.

Therefore, in the present study, we investigated N-CDH expression and NP cell phenotype under static compression and dynamic compression. Because disc organ culture maintains the disc structural integrity and disc cell extracellular environment [14–17], we performed the present study by using an *ex vivo* disc bioreactor culture system to make it at a near physiological condition.

## Materials and methods

### IVD harvest and bioreactor culture

All experimental animals were used according to the guidelines and regulations of the Ethics Committee at our hospital. The intact discs (T11-L5) with adjacent cartilage end plates were separated from healthy pigs (3–4 months old and 12–13 kg) according to a previous method [18]. Moreover, we further removed the remaining vertebral bones under a dissecting microscope. All separated discs were organ cultured and subjected to different types of compression (static compression at a magnitude of 0.4 MPa for 2 h once per day and dynamic compression at a magnitude of 0.4 MPa and a frequency of 1.0 Hz for 2 h once per day) for 7 days in the culture chambers of a mechanically active bioreactor. The noncompressed discs were used as controls. The compressive magnitude was calculated based on the disc area (Area ≈ π(WapWlat)/4, where the Wap and Wlat are the anterior–posterior and lateral widths, respectively) [19]. To decrease the damage interference to disc NP tissue caused by the mechanical overloading, the magnitude of 0.4 MPa was chosen because it is a healthy compressive magnitude [20], and is the physiological disc pressure for a person in the upright position [21]. A total of 200 ml DMEM/F12 culture medium (HyClone, U.S.A.) supplemented with 10% (v/v) FBS (Gibco, U.S.A.) and 1% (v/v) penicillin–streptomycin (Gibco, U.S.A.) was circulated at 15 ml/min. Additionally, because the sample size in one group for each experiment was relatively limited (*n*=3), each experiment was performed on the same three discs (L1/2, L2/3, and L3/4) from different animals to avoid the discrepancy between different vertebrae levels as soon as possible.

The article "Static compression down-regulates N-cadherin expression and facilitates loss of cell phenotype of nucleus pulposus cells in a disc perfusion culture" was retracted in 2024. Reasons: duplicated images; compromised peer review; concerns about the authorship.

### Alcian Blue staining assay

Discs were fixed in 4% paraformaldehyde for 48 h and then decalcified in 10% EDTA for 10–15 days. Then, the discs were processed through dehydration, embedding, and section. The 5-μm-thick cross-sections were stained by the Alcian Blue solution to investigate the proteoglycan content and distribution within the NP region. All sections were observed under a light microscope (Olympus BX51, Japan). The staining intensity was quantitated using the ImagePro Plus software (version 5.1, Media Cybernetics, Inc.)

### Real-time PCR analysis

The central NP tissue samples were isolated after culture. Then, the total RNA was extracted using the TRIzol reagent (Invitrogen, U.S.A.). After RNA quality and concentration were measured using the Nanodrop ND-1000 Spectrophotometer (Nanodrop Technologies, U.S.A.), 1 μg RNA was synthesized into cDNA. Then, the real-time PCR was performed in triplicate using SYBR Green Mix (Toyobo) together with primers (Table 1) and cDNA. The thermal cycling for PCR reaction was as follows: 3 min at 95°C, followed by 40 amplification cycles of 20 s at 95°C, 10 s at 56°C, and 15 s at 72°C. β-actin was used as an internal reference. The relative expression of target genes was analyzed using the method of 2^―ΔΔ*C*^_t_.

**Table 1:** Primers of target genes

Gene	Source	Accession number	Forward (5′–3′)	Reverse (5′–3′)
*GAPDH*	Pig	NM_001206359.1	ACCTCCACTACATGGTCTACA	ATGACAAGCTTCCCGTTCTC
*Aggrecan*	Pig	NM_001164652.1	CGTGGTCCAGCACTTCTAAA	AGTCCACTGAGATCCTCTACTC
*Collagen II*	Pig	XM_001925959.4	CCGGGTGAACGTGGAGAGACTG	CGCCCCCACAGTGCCCTC
*N-CDH*	Pig	XM_013996117.1	AACAGCAACGACGGCTTAGT	GACTGAGGTGGGTGCTGAAT
*Brachyury*	Pig	XM_001928144.4	GCCTCGAATCCACATCGTGA	TCACCGCTATGAACTGGGTC
*Laminin*	Pig	XM_005667736.2	ACGTGGTTGGAAGAAAGTGC	GACGGGATCACAGAAAGCAT
*Keratin 19*	Pig	XM_003131437.3	GGCAGAACCAGGAGTACCAG	GCCTTGATGATGGTCAGGTT

### Immunohistochemistry staining

The prepared tissue sections were processed through dewaxing, antigen retrieval, and inactivation of endogenous peroxidase. Then, they were incubated overnight at 4°C with primary antibodies (aggrecan: Novus, NB120-11570, diluted 1:200; collagen II: Abcam, ab34712, diluted 1:200) and corresponding HRP-conjugated secondary antibodies (goat antimouse IgG and goat antirabbit IgG, ZSGB-BIO, China, diluted 1:200) for 2 h at 37°C. After color development with diaminobenzidine (DAB), the sections were counterstained with Hematoxylin. The positive staining was observed under a light microscope (Olympus BX51) and quantitated using the ImagePro Plus software (version 5.1, Media Cybernetics, Inc.) to calculate the staining intensity.

The article "Static compression down-regulates N-cadherin expression and facilitates loss of cell phenotype of nucleus pulposus cells in a disc perfusion culture" was retracted in 2024. Reasons: duplicated images; compromised peer review; concerns about the authorship.

### Western blotting assay

Briefly, after the total protein was extracted using RIPA solution (Beyotime, China) with frequent agitation for 20 min and protein concentration was measured using a BCA chemical kit (Beyotime, China), equal amount of protein samples in each group was separated using SDS/PAGE and transferred on to the PVDF membrane. Then, the PVDF membrane was incubated overnight at 4°C with the primary antibodies (N-CDH, Abcam, ab18203, diluted 1:1000; β-actin, Proteintech, 60008-1-Ig, diluted 1:2000),and corresponding HRP-conjugated secondary antibodies (goat antimouse IgG and goat antirabbit IgG, ZSGB-BIO, China, diluted 1:2000) for 2 h at 37°C. Protein bands in the PVDF membrane were developed using a SuperSignal West Pico Trial Kit (Thermo, U.S.A.). The gray value of protein bands was analyzed using the ImageJ software (National Institutes of Health, U.S.A.). Protein expression of the target molecule was expressed as the ratio of the gray value of target molecule to that of β-actin.

### Biochemical content measurement

After culture, the central NP tissues were isolated and divided into two approximately equal parts. One part of NP samples were lyophilized for 24 h and digested with papain for 24 h at 60°C. Then, the glycosaminoglycan (GAG) content was calculated using the dimethyl methylene blue (DMMB) method [22]. Another part of NP samples were immediately weighted for the wet weight and then the hydroxyproline (HYP) content was calculated using a commercial HYP measurement kit (Nanjing Jiancheng, China).

### Statistics

All data expressed as the mean ± S.D. were analyzed using SPSS 13.0 software. Each experiment was performed in triplicate. The statistical difference was analyzed using one-way ANOVA, followed by an LSD post hoc test to compare between two groups. A *P*-value<0.05 indicated a significant difference.

## Results

### N-CDH expression in the static compression and dynamic compression groups

Because N-CDH is indicated to have an important role in keeping the healthy disc NP biology [12], we investigated its expression under static and dynamic compressions. Results showed that both gene (Figure 1A) and protein (Figure 1B) expression of N-CDH in the static compression group were down-regulated compared with the dynamic compression. Moreover, N-CDH expression in the control group was higher than the static compression group and lower than the dynamic compression group.

The article "Static compression down-regulates N-cadherin expression and facilitates loss of cell phenotype of nucleus pulposus cells in a disc perfusion culture" was retracted in 2024. Reasons: duplicated images; compromised peer review; concerns about the authorship.

**Figure 1:** Static compression down-regulated N-CDH expression in porcine disc NP cells compared with dynamic compression (**A**) RT-PCR analysis of *N-CDH* gene expression. *GAPDH* was used as the reference gene. (**B**) Western blotting analysis of N-CDH protein expression. Data are expressed as the means ± S.D., *n*=3; ^#^ indicates a significant difference (*P*<0.05) compared with the control group; * indicates a significant difference between two groups (*P*<0.05).

### NP cell-specific markers expression in the static compression and dynamic compression groups

The normal NP cell phenotype is beneficial to the maintenance of normal disc NP cellular function. Complete loss or attenuation of a normal NP cell phenotype occurs during disc degeneration [23,24]. The present results showed that static compression significantly decreased expression of NP-specific markers (laminin, brachyury, and keratin 19) at both gene and protein levels compared with the dynamic compression and the control group. However, their expression levels in the dynamic compression group were higher than those in the control group (Figure 2).

**Figure 2:** Static compression down-regulated gene expression of NP cell-specific markers in porcine disc NP cells compared with dynamic compression *GAPDH* was used as the reference gene. Gene expression of target genes was normalized to that of GAPDH. Data are expressed as the means ± S.D., *n*=3; ^#^ indicates a significant difference (*P*<0.05) compared with the control group; * indicates significant difference between two groups (*P*<0.05).

### NP matrix macromolecules expression in the static compression and dynamic compression groups

Within the disc NP tissue, aggrecan and collagen II are two main matrix macromolecules, which are decreased during disc degeneration [25]. In this study, we also found that static compression significantly decreased their expression levels compared with the dynamic compression and the control group, whereas their expression levels in the dynamic compression group were higher than the control group, which is reflected by the real-time PCR analysis (Figure 3A) and immunohistochemical staining (Figure 3B).

**Figure 3:** Static compression decreased expression of NP matrix macromolecules in porcine disc NP cells compared with dynamic compression (**A**) RT-PCR analysis of gene expression of aggrecan and collagen II. *GAPDH* was used as the reference gene. Gene expression of target genes was normalized to that of *GAPDH*. (**B**) Immunohistochemistry staining of aggrecan and collagen II. Magnification: 200×, scale =100 μm. Data are expressed as the means ± S.D., *n*=3; ^#^ indicates a significant difference (*P*<0.05) compared with the control group; * indicates a significant difference between two groups (*P*<0.05).

The article "Static compression down-regulates N-cadherin expression and facilitates loss of cell phenotype of nucleus pulposus cells in a disc perfusion culture" was retracted in 2024. Reasons: duplicated images; compromised peer review; concerns about the authorship.

### NP matrix component content in the static compression and dynamic compression groups

We further verified the effects of compression duration on disc NP matrix components using the Alcian Blue assay that reflects proteoglycan distribution and biochemical assay that aims to analyze the GAG and HYP contents. Our results showed that Alcian Blue staining intensity in the static compression group was lower than that in the dynamic compression group and the control group, whereas it was higher in the dynamic compression group compared with the control group (Figure 4A). Additionally, biochemical components (GAG and HYP) showed a similar trend to the Alcian Blue staining intensity amongst these groups (Figure 4B).

**Figure 4:** Static compression decreased matrix component content in porcine disc NP cells compared with dynamic compression (**A**) GAG and HYP contents measurement in porcine disc NP tissue. (**B**) Alcian Blue staining of proteoglycan content within the porcine disc NP tissue. Magnification: 200×, scale =100 μm. Data are expressed as the means ± S.D., *n*=3; ^#^ indicates a significant difference (*P*<0.05) compared with the control group; * indicates a significant difference between two groups (*P*<0.05).

## Discussion

Mechanical load plays an important role in disc development and degeneration through affecting disc cell’s biological function [26]. Static compression and dynamic compression are two common mechanical stimuli experienced by the IVD during daily activities [7]. Previous studies generally reached a consensus that static compression often facilitates disc catabolic metabolism and induces degeneration-like changes compared with the dynamic compression [6]. However, the underlying mechanisms were unknown. N-CDH is previously indicated to have a positive role in maintaining normal NP-specific phenotype [12,13]. Our study demonstrated that static compression significantly down-regulated the expression of N-CDH and NP-specific markers (brachyury, laminin, and keratin 19) and attenuated disc NP matrix biosynthesis compared with the dynamic compression. The present study suggests a relationship between N-CDH expression, NP-specific phenotype, and NP matrix biosynthesis under static and dynamic compressions.

The article "Static compression down-regulates N-cadherin expression and facilitates loss of cell phenotype of nucleus pulposus cells in a disc perfusion culture" was retracted in 2024. Reasons: duplicated images; compromised peer review; concerns about the authorship.

Cadherins are membrane-spanning molecular complexes: the extracellular regions function in adhesive recognition [27] and the cytoplasmic tails interact with certain proteins to mediate intracellular signaling and actin cytoskeleton [28]. N-CDH is first found to participate in the neural crest development and neuronal connection formation [8]. Several recent studies have also demonstrated the existence of N-CDH in disc NP tissue [12,13,29]. Additionally, as a NP cell-specific marker [10], N-CDH mediated signaling can promote maintenance of NP-specific phenotype and NP matrix biosynthesis *in vitro* [12,13]. In light of the loss of NP-specific phenotype and accelerated NP matrix degradation during disc degeneration, those previous studies [10,12,13,29] on N-CDH indicate that N-CDH expression is important to retain NP-specific phenotype and NP matrix biosynthesis, which may be a biological strategy for preservation of healthy disc NP tissues or retarding disc degeneration.

In line with the previous studies [6,7] we found that static compression caused NP matrix catabolic metabolism compared with the dynamic compression, which was reflected by the decreased matrix molecules (aggrecan and collagen II) expression and matrix components (GAG and HYP) content. Meanwhile, NP-specific markers were also down-regulated by static compression compared with the dynamic compression. These findings further verify that static compression is more harmful to healthy disc cell biology than the dynamic compression. The present study reported for the first time in a disc organ culture that static compression decreased N-CDH expression compared with the dynamic compression. In light of the previous reported advantageous effects of N-CDH on the maintenance of NP-specific phenotype and NP matrix biosynthesis, the present findings suggest that alleviation of N-CDH-mediated signaling may partly contribute to mechanical load-induced degenerative changes of the disc NP tissue. However, additional experiments, such as enhancing N-CDH expression or silencing N-CDH expression, are necessary to further confirm this point and investigate the underlying signaling transduction in the future.

Several limitations also existed in the present study. First, the immature porcine disc NP tissue has a high content of notochordal cells [30]. This differs from the adult human disc NP tissue, which may limit present study’s stringency in imitating the mechanobiology of the adult disc. Second, though the present conclusion was based on the previous studies, experiment of enhancing N-CDH expression or silencing N-CDH expression was not performed to confirm the effects of N-CDH on maintaining NP-specific phenotype and the resulting NP matrix biosynthesis under static and dynamic compressions. Third, an animal *in vivo* study cannot performed to further confirm our results due to the lack of appropriate experiment platforms.

The article "Static compression down-regulates N-cadherin expression and facilitates loss of cell phenotype of nucleus pulposus cells in a disc perfusion culture" was retracted in 2024. Reasons: duplicated images; compromised peer review; concerns about the authorship.

In conclusion, static compression simultaneously down-regulates the expression of N-CDH and NP cell-specific markers and declines NP matrix biosynthesis compared with dynamic compression. In light of the previously reported advantageous effects of N-CDH on NP-specific phenotype and NP matrix biosynthesis, the present study indirectly suggests that down-regulation of N-CDH may be responsible for NP-specific phenotype alteration and NP matrix degeneration under the static compression.

## Abbreviations

GAG: glycosaminoglycan
GAPDH: glyceraldehyde-3-phosphate dehydrogenase
HRP: horseradish peroxidase
HYP: hydroxyproline
IVD: intervertebral disc
LBP: low back pain
NP: nucleus pulposus
N-CDH: N-cadherin
RT-PCR: reverse transcription-polymerase chain reaction
